# MicroRNA-182 modulates chemosensitivity of human non-small cell lung cancer to cisplatin by targeting PDCD4

**DOI:** 10.1186/1746-1596-9-143

**Published:** 2014-07-10

**Authors:** Fang-ling Ning, Feng Wang, Mian-li Li, Ze-shun Yu, Yan-zhang Hao, Shao-shui Chen

**Affiliations:** 1 Department of Oncology, Binzhou Medical College Affiliated Hospital, 661#, Yellow-River Second Street, 256603 Binzhou, Shandong Province, China

**Keywords:** miRNA, PDCD4, miR-182, Chemosensitivity, A549, NSCLC

## Abstract

**Abstract:**

**Background**

Overexpression of microRNA-182 (miR-182) is found in various human cancers, including non-small cell lung cancer (NSCLC). Our aim is to investigate the association of miR-182 expression with the sensitivity of NSCLC to cisplatin.

**Methods**

TaqMan RT-PCR or Western blot assay was performed to detect the expression of mature miR-182 and programmed cell death 4 (PDCD4) protein. miR-182 and (or) PDCD4 depleted cell lines were generated using miR-182 inhibitor and (or) siRNA. The viabilities of treated cells were analyzed using MTT assay.

**Results**

The expression level of miR-182 in A549 cell line was significantly higher than that in NHBE cell line (p < 0.01). Transfection of miR-182 inhibitor induced sensitivity of A549 cells to cisplatin. A549 cells transfected with PDCD4 siRNA became more resistant to cisplatin therapy. We found an increase PDCD4 protein level following the transfection of miR-182 inhibitor using Western blot analysis. In addition, the enhanced growth-inhibitory effect by miR-182 inhibitor was weakened after the addition of PDCD4 siRNA.

**Conclusions**

The results of the present study demonstrated that overexpression of miR-182 may involve in chemoresistance of NSCLC cells to cisplatin by down-regulating PDCD4.

**Virtual Slides:**

The virtual slide(s) for this article can be found here: http://www.diagnosticpathology.diagnomx.eu/vs/1793467320130186

## Background

Lung cancer is the most common cancer in the world, with a survival rate of 15% [1]. Approximately 1.6 million cases of lung cancer have occurred in 2008, of which 80% were non-small cell lung cancer (NSCLC). Surgical resection is known as the most effective treatment for NSCLC, however, due to the fact that most diagnoses were confirmed in an advanced stage, only a few patients can be cured by surgical treatment. Patients with NSCLC are mostly treated with platinum-based chemotherapy. However, the development of chemoresistance is a major obstacle limiting successful treatment [2]. Methods for improving chemotherapy and reducing chemoresistance are accordingly of great interest in lung cancer chemotherapy [3,4].

MicroRNAs (miRNAs) are small non-coding RNAs of 20 ~ 22 nucleotides. It represses gene expression through interaction with 3′untranslated regions (UTRs) of mRNAs. miRNAs are predicted to target over 50% of all human protein-coding genes, enabling them to have numerous regulatory roles in many physiological and developmental processes, including development, differentiation, apoptosis and proliferation, through imperfect pairing with target mRNAs of protein-coding genes and the transcriptional or post-transcriptional regulation of their expression [5,6]. miR-182 is one of the miRNAs often seen upregulated in cancers. Several studies have reported miR-182 to be upregulated in NSCLC [7]. Furthermore, miR-182 functions as an oncomiR to enhance cancer cell proliferation [8,9]. Recent studies indicated that miR-182 plays an important role in drug resistance. Husted et al. found that miR-182 was consistently upregulated in the multidrug resistant Ehrlich ascites tumor cells [10]. Therefore, we hypothesized that the up-regulation of miR-182 may be related to chemotherapy resistance in NSCLC, but the molecular mechanism remains unclear.

As an important tumor suppressor, programmed cell death 4 (PDCD4) influences transcription and translation of multiple genes, and modulates different signal transduction pathways. However, the upstream regulation of this gene is largely unknown. Until now, the mainly identified miRNA that directly targets PDCD4 is microRNA-21 (miR-21). MiR-21 has been found to negatively regulate PDCD4 expression in breast cancer, colorectal cancer, and ovarian cancer [11-13]. However, other potential PDCD4-targeting miRNAs remains to be defined. We speculate that miR-182 may play an important role in chemoresistance of A549 cells by down-regulating the PDCD4.

## Methods

### Cell line

The Human Research Ethics Committee of Binzhou Medical College Affiliated Hospital approved this study. The human lung adenocarcinoma cell line A549 was purchased from the Cell Bank of Chinese Academy of Sciences (Shanghai, China). A549 cell line was cultured in DMEM containing 10% fetal bovine serum (Gibco®, Invitrogen, Carlsbad, CA, USA), 100 units/ml penicillin, and 100 μg/ml streptomycin at 37°C in a 5% CO2 humidified incubator to the log phase of proliferation before harvesting the cells. Normal human bronchial epithelial cells (NHBE) (Clonetics™) were maintained in a culture medium according to the protocol provided by Clonetics™.

### Drugs and reagents

Cisplatin was purchased from QiLu Pharmaceutical (Jinan, China). MiR-182 inhibitor, PDCD4 siRNA, and their negative control oligonucleotides were obtained from Shanghai GeneChem Co., Ltd (Shanghai, China). These were used to transfect A549 cells using Lipofectamine™ 2000 (Invitrogen, Carlsbad, CA, USA) according to the instructions provided by the manufacturer. Monoclonal rabbit anti-human PDCD4 antibody (Cell Signaling Technology, Inc., Beverly, MA, USA) was used for Western blot analysis.

### MTT assay

Cells transfected with miR-182 inhibitor or siRNA-PDCD4 were seeded into 96-well plates at 6*10^3^ cells/well and allowed to grow overnight, and then were treated with different concentrations of cisplatin. After 24 h of treatment, 20ul of 5 mg/ml MTT reagent (Sigma-Aldrich, St. Louis, MO, USA) was added and incubated in the dark for 4 h. The absorbance of the plate was measured in a microplate reader at a wavelength of a 570-nm reference (BMG Lab Technologies, Germany), and the results were expressed as the percentage of absorbance relative to untreated controls. Each treatment was carried out in triplicate.

### Real-time quantitative reverse transcription-PCR for miRNA expression and mRNA expression

For miRNA expression detection, reverse transcription (RT) reaction was performed with PrimeScript® RT reagent Kit (TAKARA BiotechnologyCO., LTD., Dalin, China) and realtime quantitative RT-PCR (qRT-PCR) was performed using SYBR® Premix Ex Taq™ II (TAKARA Biotechnology CO., LTD., Dalin, China) on the basis of the protocol provided by the manufacturer. For mRNA expression detection, reverse transcription reaction was performed with PrimeScript® RT reagent Kit (TAKARA Biotechnology CO., LTD., Dalin, China) and RT-PCR (qRT-PCR) was performed using SYBR® Premix Ex Taq™ II (TAKARA Biotechnology CO., LTD., Dalin, China). The designed PCR primers were as follows: PDCD4 forward primer, 5’-GGCCTCCAAGGAGTAAGACC-3’; PDCD4 reverse primer, 5’-AGGGGTCTACATGGCAACTG-3’; GAPDH forward primer, 5’-AAGGGAAGGTTGCTGGATAGG-3’; GAPDH reverse primer, 5’-CACATCCACCTCCTCCACATC-3’. The expression of the target miRNA was normalized relative to that of the internal control, U6 and the expression of the target gene was normalized relative to the expression of glyceraldehyde-3-phosphate dehydrogenase (GAPDH), which was used as an internal control. Data were analyzed according to the comparative Ct method also referred to as the 2^-ΔΔCT^ method.

### Western blot assay

The proteins were resolved on an SDS denaturing polyacrylamide gel and then transferred onto a nitrocellulose membrane. Antibody to PDCD4 or GAPDH was incubated with the membranes overnight at 4°C. The membranes were washed and incubated with horseradish peroxidase (HRP)-conjugated secondary antibodies. Protein expression was assessed by enhanced chemiluminescence and exposure to chemiluminescent film. LabWorks™ Image Acquisition and Analysis Software (UVP, Upland, CA) were used to quantify the band intensities. All the antibodies were purchased from Abcam (Cambridge, MA).

### Statistical analysis

All the experiments were carried out in triplicate. The quantitative values were expressed as mean ± standard deviation (SD), and the hypothesis test for significance between two groups utilized the Student’s *t* test. Statistical significance was set as p <0.05.

## Results

### MiR-182 was upregulated in human lung adenocarcinoma cell line A549

To define the role of miR-182 in human lung cancer tumorigenesis, we compared the expression levels of miR-182 in human lung cancer cell line A549 and NHBE cell line (normal human bronchial epithelial cells) by qRT-PCR. The expression level of miR-182 in A549 was significantly higher than that in NHBE cell line (p < 0.01, Figure 1).

**Figure 1:** MiR-182 was up-regulated in A549 cell line compared to that in NHBE cell line (p < 0.01).

### Transfection of miR-182 inhibitor induced sensitivity of A549 cells to cisplatin

To further assess the effect of miR-182, we transfected miR-182 inhibitor and its negative control oligonucleotides into A549 cells. Transfection of cells with miR-182 inhibitor suppressed miR-182 level compared with the control cells (shown in Figure 2). The MTT assay showed that the miR-182-suppressed cells were significantly more sensitive to the therapy of cisplatin than control cells (shown in Figure 3).

**Figure 2:** **Transfection of miR-182 inhibitor and its negative control oligonucleotides (NC) into A549 cells.** qRT-PCR showed significant under-expression of miR-182 in the transfected cells compared with control cells.

**Figure 3:** MTT assay revealed that the anti-tumour effects cisplatin in the miR-182 downregulated cells were significantly profound than in control cells (*P <0.05). Data are mean ± SD of three experiments.

### PDCD4 was a target of miR-182 and responsible for the miR-182-induced resistance in A549 cells

We transfected A549 cells with miR-182 inhibitor or a scrambled miR-182 inhibitor control. The PDCD4 mRNA level was overexpression in miR-182-suppressed cells compared with controls (shown in Figure 4a). We examined the protein levels of PDCD4 following the transfection of miR-182 inhibitor in A549 cells by Western blot analysis and found that cells transfected with miR-182 inhibitor showed an increase PDCD4 protein expression (shown in Figure 4b). Down regulation of PDCD4 expression by siRNAs, A549 cells became more resistant to the therapy of cisplatin (shown in Figure 5). In addition, the enhanced growth-inhibitory effect by the miR-182 inhibitor transfection was weakened after the addition of PDCD4 siRNA (shown in Figure 5).

**Figure 4:** **Evaluation of PDCD4 in A549cells transfected with miR-182 inhibitor and its negative control oligonucleotides (NC). A.** qRT-PCR showed significant upregulation of PDCD4 mRNAs in the transfected cells. **B.** Western blot analysis demonstrated significant overexpression of PDCD4 proteins in the transfected cells (*P < 0.05). Data are mean ± SD of three experiments.

**Figure 5:** **Changes in anti-tumour effects of the cisplatin after transfection of anti-miR-182 and/or siRNA against PDCD4 in A549 cells.** The MTT assay indicated a weaker anti-tumour effect of cisplatin following transfection of PDCD4 siRNA, and the enhanced growth-inhibitory effect by anti-miR-182 transfection was also weakened after the addition of PDCD4 siRNA (*P <0.05).

## Discussion

Although chemotherapeutic agents are widely used in the treatment of lung cancer, their efficacy is often limited by the existence or development of chemoresistance. As one of the first-line chemotherapeutic agents for the treatment of NSCLC, cisplatin is a platinum-based compound that forms intra- and inter-strand adducts with DNA [14,15]. Despite tremendous efforts, cisplatin treatment often results in the development of drug resistance, leading to therapeutic failure, and the molecular mechanisms leading to cisplatin chemoresistance are poorly understood. Factors that enhance the sensitivity of NSCLC cells to cisplatin may highlight predictive biomarkers or targets for therapy.

MiRNAs are thought to function as either tumor suppressors or oncogenes though target oncogenes or tumor suppressor genes during tumorigenesis and development of cancers [16-18]. miR-182 has been regarded as an oncogene in most contexts. In a cohort of 253 glioma patients, high miR-182 expression was found to be a negative prognostic factor [19]. In melanoma cell lines, Segura and coworkers showed that high miR-182 expression stimulated migration and survival. The same group treated liver metastases in mice with anti -miR-182 and obtained a lower tumor burden and a lower mir-182-level than in untreated mice [20]. Also in breast tumors and cervical cancers miR-182 seems to have an oncogenic impact [21,22]. Previously, Wang M et al. found that miR-182 was markedly upregulated in human lung cancer cells. They conducted MTT and colony formation assays to further evaluate the effect of miR-182 on lung cancer cell growth, and they performed transwell and wound healing assays to evaluate its role in regulating invasion and migration activity. Their results demonstrate that miR-182 acts as an oncogene in lung cancer [9].

Previous studies demonstrated that the acquired drug resistance of cancer cells is related to deregulation of miRNAs such as miR21, miR-503, miR-181a and miR-620 [23-25]. In the present study, to explore whether the unregulated oncogene miR-182 was involved in the NSCLC cells resistant to cisplatin, we transfected miR-182 inhibitor and its negative control oligonucleotides into A549 cells. Then MTT assay showed that the miR-182-suppressed cells were significantly more sensitive to the therapy of cisplatin than control cells, indicating that overexpression of miR-182 may involve in chemoresistance of NSCLC cells to cisplatin.

In NSCLC tissues, many onco-miRs/tumor suppressor-target or tumor suppressor-miRs/onco-target pathways have been demonstrated to participate in the tumorigenesis of lung cancer, including miR7/BCL2 axis, miR-99b/FGFR3 axis, miR-101/EZH2 axis, miR-192/RB1 axis and miR-196/HOXA5 axis [26-30]. However, miRNA/target network was so complex that more and more miRNA/target axis needs to be elucidated in lung cancer especially NSCLC. In the present study, We transfected A549 cells with miR-182 inhibitor or a scrambled miR-182 inhibitor control. The PDCD4 mRNA and protein were overexpression in miR-182-suppressed cells compared with controls, indicating that miR-182 was a negative regulator of PDCD4. Furthermore, we found that when down regulated of PDCD4 expression by siRNAs, A549 cells became more resistant to the therapy of cisplatin. In addition, the enhanced growth-inhibitory effect by the miR-182 inhibitor transfection was weakened after the addition of PDCD4 siRNA, suggesting that PDCD4 was responsible for the miR-182-induced resistance to cisplatin. These results established that miR-182 transfer in combination with cisplatin therapy may be a target to reverse chemotherapeutic resistance. In addition, further research is needed to investigate whether the expression level of miR-182 in tumor tissue and plasma might be used as a biomarker to predict platinum based chemotherapy response in patients with NSCLC.

## Conclusion

In conclusion, the results of the present study demonstrates that overexpression of miR-182 may involve in chemoresistance of NSCLC cells to cisplatin by down-regulating PDCD4. This finding suggests that inhibition of miR-182 may be a useful therapeutic strategy for NSCLC treatment.

## Competing interests

The authors declare that they have no competing interests.

## Authors’ contributions

FLN, FW and SSC: conceived of the study, and participated in its design and coordination and helped to draft the manuscript. FLN, FW, MLL, ZSY and YZH: carried out part of experiments and wrote the manuscript. FLN, FW and MLL performed the statistical analysis. All authors read and approved the final manuscript.
